This article has been retracted.

# A Matrine Derivative M54 Suppresses Osteoclastogenesis and Prevents Ovariectomy-Induced Bone Loss by Targeting Ribosomal Protein S5

**DOI:** 10.3389/fphar.2018.00022

**Published:** 2018-01-30

**Authors:** Zhi Xin, Cui Jin, Liu Chao, Zhang Zheng, Cao Liehu, Pan Panpan, Weng Weizong, Zhai Xiao, Zhao Qingjie, Hu Honggang, Qin Longjuan, Chen Xiao, Su Jiacan

**Affiliations:** ^1^Graduate Management Unit, Shanghai Changhai Hospital, Second Military Medical University, Shanghai, China; ^2^School of Pharmacy, Second Military Medical University, Shanghai, China; ^3^Department of Orthopedics, Shanghai Changhai Hospital, Second Military Medical University, Shanghai, China; ^4^China-South Korea Bioengineering Center, Shanghai, China; ^5^Orthopedic Basic and Translational Research Center, Jiangyin, China

**Keywords:** RPS5, matrine derivative, RANKL, osteoclasts, AKT pathway

## Abstract

Post-menopausal osteoporosis (PMOP) is a metabolic bone disorder characterized by low bone mass and micro-architectural deterioration of bone tissue. The over-activated osteoclastogenesis, which plays an important role in osteoporosis, has become an important therapeutic target. M54 was a bioactive derivative of the Chinese traditional herb matrine. We found that M54 could suppress RANKL-induced osteoclastogenesis in bone marrow mononuclear cells and RAW264.7 cells through suppressing NF-κB, PI3K/AKT, and MAPKs pathways activity *in vitro*, and prevent ovariectomy-induced bone loss *in vivo*. Our previous study has proved that ribosomal protein S5 (RPS5) was a direct target of M19, based on which M54 was synthesized. Thus we deduced that M54 also targeted RPS5. During osteoclastogenesis, the RPS5 level in RAW264.7 cells was significantly down-regulated while M54 could maintain its level. After RPS5 was silenced, the inhibitory effects of M54 on osteoclastogenesis were partially compromised, indicating that M54 took effects through targeting RPS5. In summary, M54 was a potential clinical medicine for post-menopause osteoporosis treatment, and RPS5 is a possible key protein in PMOP.

## Introduction

Post-menopausal osteoporosis (PMOP) is the most common degenerative bone disease, affecting millions of post-menopausal women (Del Puente et al., 2015), and it is also the most common primary osteoporosis characterized by decreased bone density and increased fracture risks (Wu et al., 2015). Bone is continuously remodeled in life by the interaction between bone resorbing osteoclasts with bone forming osteoblasts (Chen et al., 2016). Over-activation of osteoclasts is a major cause of osteoporosis (Jakob et al., 2015). Osteoclasts play an important role in bone destruction in common erosive bone diseases, such as PMOP, rheumatoid arthritis, and periodontitis (Zhang et al., 2015). In these conditions, increased production of the receptor activator of nuclear factor-κB (NF-κB) ligand (RANKL) and pro-inflammatory cytokines including IL-6, TNF-α which activate bone resorption by osteoclasts (Walsh and Choi, 2014). Signaling is regulated by recruitment of TNF receptor-associated factors (TRAFs) and results in activation of transcription factors including AKT, MAPK, NF-κB, c-Fos, and NFATc1 in osteoclast precursors (Nakashima et al., 2011).

Traditional Chinese herbs provide abundant sources for anti-osteoporosis medicine (Li et al., 2014). Matrine is the major component of traditional Chinese herb Sophora flavescens Ait and exhibited significant anti-inflammatory and anti-fibrotic pharmacological effects (Qian et al., 2015; Li J. Z. et al., 2016; Sun et al., 2016). M54 was produced based on matrine, and exhibited better anti-inflammatory effect than matrine itself, which indicated the promising anti-osteoclastogenesis effect of M54. Besides, RPS5 was proved to be a direct target of matrine derivative, referred to the inhibitory effect on liver fibrosis (Xu et al., 2014).

The purpose of our study is to investigate the roles of RPS5 in osteoclastogenesis and the effects of M54 on bone loss in ovariectomized mice.

## Materials and Methods

### Reagents

Reagent M54 (M54, **Figure 1A**) was supplied by Prof. Hu from the School of Pharmacy, Second Military Medical University. Briefly, sophocarpine was transformed into thiosophocarpine in high yield by treatment with Lawesson’s reagent. Then, M19 was synthesized by reaction of thiosophocarpine with NH_2_CH_3_. M54 was synthesized by reaction of M19 with CO_2_ and benzyl bromide. M54 was dissolved in ddH_2_O for use *in vitro* and dissolved in normal saline as vehicle for use *in vivo*. DMEM and fetal bovine serum (FBS) was obtained from Hyclone (Logan, UT, United States). Penicillin–streptomycin was obtained from Sangon Biotech (Shanghai City, IL, United States). Soluble recombinant mouse RANKL and M-CSF were purchased from R&D (R&D Systems, Minneapolis, MN, United States). Tartrate-resistant acid phosphatase (TRAP) Kit was obtained from Sigma-Aldrich (St. Louis, MO, United States). RAW264.7 cells were purchased from Central Plains Cell Institute (Shanghai, China).

**FIGURE 1:** M54 inhibits RANKL-induced osteoclast differentiation and bone resorption *in vitro*. **(A)** Chemical structure of M54 and the synthesis process. **(B)** Formation of TRAP-positive cells from BMMCs and the quantification of formed osteoclasts. **(C)** Formation of TRAP-positive cells from RAW264.7 cells and the quantification of formed osteoclasts. **(D)** The resorption area on the bone biomimetic synthetic surface was quantified by image analysis (^∗^*P* < 0.05, ^∗∗^*P* < 0.01, ^∗∗∗^*P* < 0.001).

### *In Vitro* Osteoclastogenesis Assay

The 8-week-old C57BL/6 mice were used to collect bone marrow mononuclear cells (BMMCs) (Guan et al., 2015). The BMMCs were cultured in DMEM low glucose medium, FBS, and penicillin–streptomycin mixture until the number is enough. Following, M-CSF (20 ng/ml) and RANKL (50 ng/ml) were used for osteoclast induction, which was treated with M54 (1, 2, 4 μM) or vehicles for 7 days. TRAP staining was carried out according to the manufacturer’s instructions for osteoclasts detection. RAW264.7 cells were also induced with M-CSF (20 ng/ml) and RANKL (50 ng/ml), and treated with M54 (1, 2, 4 μM) or vehicles for 7 days before TRAP staining. Cells were counted as osteoclasts if they were TRAP^+^ multinucleated (nuclei > 5 for BMMCs and nuclei > 3 for RAW264.7 cells) (Wu et al., 2012; Ouyang et al., 2014).

### *In Vitro* Bone Resorption Pit Assay

A hydroxyapatite-coated plate (Corning, Lowell, MA, United States) was used for osteoclast bone resorption effects detection (Zeng et al., 2017). RAW264.7 cells (1 × 10^4^ cells/well) were cultured in the plate with 50 ng/ml RANKL for osteoclast induction. The cells were treated with varying concentrations of M54 (1, 2, 4 μM) or vehicles. Medium change was carried out on day 3. The plate was cleaned with 10% bleach solution and air dried for 3–5 h at room temperature, after 7 days. The pictures of pits at the well bottom were taken with light microscope (OLYMPUS, IX71), and the pit areas were quantified with software Image-Pro Plus 6.0.

### Western-Blot Analysis

RAW264.7 cells and lentivirus infected RAW264.7 cells were used for immunoblot analysis. For osteoclastogenesis evaluation, the osteoclastogenesis-related markers Cathepsin K, CTR, MMP-9, NFATc1, and TRAP were detected. To define the mechanism of M54 affects osteoclastogenesis, RPS5 expression and the phosphorylation of pathway key protein AKT, P65, IκB, ERK, JNK, and P38 were detected.

M-PER mammalian protein extraction reagent (Pierce, IL, United States) was used to extract the total protein. The membranes were cut according to the molecular size of the target protein and re-incubated with primary antibodies but using the same loading control. Equal amounts of protein (10 μg per lane) estimated by a bicinchoninic acid (BCA) protein assay kit (Pierce) were loaded onto (11%) SDS-PAGE gels and transferred onto nitrocellulose membranes. The primary antibody included mouse anti-Cathepsin K (1:500), anti-CTR (1:200), anti-MMP-9 (1:400), anti-NFATc1 (1:250), anti-TRAP (1:350), anti-RPS5 (1:150), anti-AKT (1:250), anti-P-AKT (1:400), anti-P65 (1:350), anti-P-P65 (1:500), anti-IκBa (1:350), anti-P-IκBa (1:500), anti-anti-ERK (1:200), anti-P-ERK (1:400), anti-JNK (1:500), anti-P-JNK (1:400), anti-P38 (1:300), anti-P-P38 (1:300), and anti-beta actin (1:1000) (Santa Cruz, CA, United States). The following secondary anti-body was HRP-conjugated anti-mouse/rabbit antibody (Santa Cruz, CA, United States). Finally, the results were detected by chemiluminescence.

### Preparation of Lentivirus and Lentivirus Infection

RPS5 knockdown lentivirus were prepared to study the effects of RPS5 on osteoclastogenesis. A siRNA sequence (5′-GCTCATGACTGTGCGAATT-3′) of RPS5 was chosen to construct the RPS5 silence vector pSIH1-shRNA-RPS5 plasmid. At the same time, an invalid siRNA sequence (5′-GAAGCCAGATCCAGCTTCC-3′) was used to construct another vector pSIH-NC for negative control (NC). The vectors were all marked with green fluorescence marker GFP. Then the plasmids were used to transfect 293TN cells to package and product recombinant lentivirus Lv-shRNA-RPS5 and Lv-NC.

RAW264.7 cells were cultured into 6-well plates, and the cell culture methods were still as described before. After 1-day culture, the prepared lentivirus was added into wells with a multiplicity of infection (MOI) of 20 to infect cells. To determine the genetic intervention efficiency, the cells were collected after 72 h for RPS5 protein Western-blot examination.

### Animal Preparation

The animal model protocols of this study were approved by the standards of the Ethics Committee of Second Military Medical University and conformed to the U.S. National Institutes of Health guidelines for use of animals in research. Female 8-week-old C57BL/6 mice were purchased from Slack (Shanghai, China), and all the animal experiments were implemented in the Specific Pathogen Free (SPF) animal laboratory of Changhai Hospital [certification: SCXK (Shanghai) 2007-0003].

### Ovariectomy (OVX) Animal Model

The female 8-week-old mice were divided into three groups with 6 per group: sham group, ovariectomized (OVX) mice treated with vehicle and OVX mice treated with M54. The OVX surgery were carried out as previously described (Zhou et al., 2016). After Sham or OVX surgery, the treated mice were given intraperitoneally (i.p.) of M54 (250 mg/kg) which was the highest affordable dose for the mice, and the OVX mice were given intraperitoneally of same volume of normal saline. The injection was carried out every day for 6 weeks. Following, the mice were anesthetized with chloral hydrate. Serum was collected for biochemistry examination, and bilateral femurs were excised and fixed in 4% paraformaldehyde solution for histologic and Micro-CT analysis.

### Histomorphometric Examination

The left femurs were fixed in 4% paraformaldehyde solution for 4 days, and then decalcified by 10% tetracycline-EDTA aqueous solution for 2 weeks. After decalcification, the femurs were paraffin-embedded to prepare 4-mm sections for hematoxylin and eosin (H&E) staining and TRAP staining. Bone trabecula was observed in H&E-stained sections, and the osteoclasts were observed in TRAP-stained sections. Image-Pro Plus 6.0 was used for compute trabecular area, and count the number of osteoclasts in the region of the metaphysis.

### Micro-CT Analysis

The right femurs were scanned at 9 μm resolution in a micro-CT instrument (supported by Huaiyu Biological Technology Limited Company, Shanghai, China). Trabecular bone was analyzed within a volume of slices spanning a 1-mm distance, starting 0.5 mm from the bottom of the growth plate. The build-in software of micro-CT was used to reconstruct two-dimensional and three-dimensional bon structure image slices, and analyze the parameters. The measured trabecular bone parameters include total bone mineral density (BMD), bon volume fraction (BV/TV), trabecular number (Tb. N), and bone surface area expressed per unit total volume (BS/TV).

### Serum Biochemistry

Blood was collected from the left ventricular, followed with centrifugation process of 3000 r × 5 min. Serum concentration of bone resorption biomarker TRAcp5B and inflammatory cytokines IL-6 and TNF-α, were determined with ELISA kits for TRAcp5B, IL-6 and TNF-α (Anogen, Canada) according to the manufacturer’s instructions.

### Statistical Analysis

Statistical analysis was performed with the software IBM SPSS Statistics 22. The results are presented as Mean ± SD. Differences between two groups were compared with the Student’s *t*-test. Differences between more than two groups were compared with one-way ANOVA. *P* < 0.05 was regarded as statistically significant.

## Results

### M54 Inhibits RANKL Induced Osteoclastogenesis and Bone Resorption *in Vitro*

To explore the effect of M54 on osteoclastogenesis, various concentrations of M54 were used to treat BMMCs and RAW264.7 in the presence of RANKL plus M-CSF. The TRAP staining results indicated that M54 had the effect of inhibiting RANKL induced osteoclast differentiation from BMMCs (**Figure 1B**) and RAW264.7 cells (**Figure 1C**). The number of osteoclasts were significantly decreased by M54 treatment in BMMCs and RAW264.7 cells. The function of osteoclast was also detected with hydroxyapatite-coated plats. The results indicated that treatment of M54 inhibited the bone resorption function of osteoclasts (**Figure 1D**).

### M54 Promotes RPS5 Expression in RANKL-Induced Osteoclast *in Vitro*

As previous study described, matrine derivatives targeted RPS5. Western-blot was used to explore the effect of M54 on RPS5 expression in RANKL-induced osteoclast *in vitro*. The Western-blot results indicated that RPS5 expression were significantly decreased in RANKL induced group (*P* < 0.01), and M54 treatment ameliorated the change (*P* < 0.01) in a dose-dependent manner (**Figure 2A**).

**FIGURE 2:** M54 promotes RPS5 expression and suppresses PI3K/AKT, NF-κB, and MAPK pathways activity pathways. **(A)** Western-blot results of RPS5 protein expression. **(B)** Phosphorylation of AKT protein, which was associated with PI3K/AKT pathway. **(C)** Phosphorylation of P65 protein, which was associated with NF-κB pathway. **(D)** Phosphorylation of ERK, JNK, and P38 protein, which was associated with MAPK pathway. ➀RAW264.7 cells; ➁RAW264.7 cells induced with M-CSF, RANKL and PBS; ➂RAW264.7 cells induced with M-CSF, RANKL and treated with 1 μM M54; ➃RAW264.7 cells induced with M-CSF, RANKL and treated with 2 μM M54; ➄RAW264.7 cells induced with M-CSF, RANKL and treated with 4 μM M54 (^∗^*P* < 0.05, ^∗∗^*P* < 0.01 vs. ➁).

### M54 Inhibits Multiple Pathways Involved in Osteoclast Differentiation

Western-blot assays were used to detect the activities of osteoclastogenesis related pathways PI3K-AKT, NF-κB, and MAPK. The phosphorylation of the key protein of PI3K-AKT pathway AKT was significantly promoted by RANKL induction (*P* < 0.01), and M54 treatment reduced the phosphorylation significantly (*P* < 0.01) in a dose-dependent manner (**Figure 2B**). The phosphorylation of major subfamilies of NF-κB and MAPK pathways IκB, P65, ERK, JNK, and P38 were also detected. The phosphorylation of the key proteins was significantly increased (*P* < 0.01) after RANKL induction, which was significantly inhibited (*P* < 0.01) by M54 treatment (**Figures 2C,D**). These data indicated the effect of M54 to suppress PI3K-AKT, NF-κB, and MAPK pathways activation.

### M54 Inhibits Expressions of Osteoclastogenesis-Related Markers

The expressions of osteoclastogenesis-related markers were also detected by Western-blot assays. The makers included Cathepsin K, CTR, MMP-9, NFATc1, and TRAP. M54 treatment significantly (*P* < 0.01) inhibited the expression of the markers, which were increased (*P* < 0.01) by RANKL induction (**Figure 3**).

**FIGURE 3:** M54 inhibits expressions of osteoclastogenesis-related markers. Western blot and optical density analysis of expression of Cathepsin K, CTR, MMP-9, NFATc1, and TRAP with Beta actin as reference. ➀RAW264.7 cells; ➁RAW264.7 cells induced with M-CSF, RANKL and PBS; ➂RAW264.7 cells induced with M-CSF, RANKL and treated with 1 μM M54; ➃RAW264.7 cells induced with M-CSF, RANKL and treated with 2 μM M54; ➄RAW264.7 cells induced with M-CSF, RANKL and treated with 4 μM M54. The membranes were cut according to the molecular size of the target protein and reincubated with primary antibodies but using the same loading control (^∗∗^*P* < 0.01, ^∗^*P* < 0.05 vs. ➁).

### RPS5 Expression Was Regulated by Lentivirus Infection and M54 Treatment

The relationship between M54 treatment and RPS5 expression was evaluated. To make RPS5 silenced cells, lentivirus were used to infect RAW264.7 cells. After 72 h, the expression of green fluorescence marker GFP was detected to ensure that the infected efficiency of RAW264.7 cells were close to 100% (**Figure 4A**). Western-blot examination was used to confirm that RPS5 was silence with the former steps (**Figure 4B**). The results indicated that the expression of RPS5 were significantly suppressed by Lv-shRNA-RPS5, however was not affected by Lv-NC (**Figure 4B**). Thus, cells infected with Lv-shRNA-RPS5 were identified to be RPS5 silenced cells, and cells infected with Lv-NC were set as normal cells. Two series of experiments with RANKL induction and M54 treatment (1 μM) were conducted in both cells with RPS5 silencing (➃, ➄, and ➅) or without PRS5 silencing (➀, ➁, and ➂). As shown in **Figure 4C**, RANKL induction significantly suppressed the RPS5 expression (➁ vs. ➀, ➄ vs. ➃, *P* < 0.01); the M54 treatment ameliorated the effects of RANKL induction (➂ vs. ➁, ➅ vs. ➄, *P* < 0.01).

**FIGURE 4:** RPS5 partially ameliorate the effect of M54. **(A)** Fluorescence of cells infected with lentivirus after 72 h. a, b was infected with Lv-NC and c, d was infected with Lv-shRNA-RPS5. **(B)** Detection of intracellular RPS5 protein expression, MOI = 20. **(C)** RPS5 expression in lentivirus infected RAW264.7 with or without M54 treatment (1 μM). **(D)** Phosphorylation of AKT and C-FOS. ➀RAW264.7 cells infected with Lv-NC; ➁RAW264.7 cells infected with Lv-NC and induced with M-CSF, RANKL and PBS; ➂RAW264.7 cells infected with Lv-NC, induced with M-CSF, RANKL and treated with 4 μM M54; ➃RAW264.7 cells infected with Lv-shRNA-RPS5; ➄RAW264.7 cells infected with Lv-shRNA-RPS5 and induced with M-CSF, RANKL and PBS; ➅RAW264.7 cells infected with Lv-shRNA-RPS5, induced with M-CSF, RANKL and treated with 4 μM M54 (^∗∗^*P* < 0.01, ^∗^*P* < 0.05 vs. ➁).

### RPS5 Silencing Partially Ameliorates the Effects of M54 on PI3K/ATK and MAPK Pathways

The above results indicated that M54 inhibited the expression of osteoclastogenesis related pathways PI3K-AKT, NF-κB, and MAPK, and osteoclastogenesis related markers Cathepsin K, CTR, MMP-9, NFATc1, and TRAP. Lentivirus infected RAW264.7 cells were used to investigate the role of RPS5 on osteoclatogenesis. Two series of experiments with RANKL induction and M54 treatment (1 μM) were conducted in both cells with RPS5 silencing (➃, ➄, and ➅) or without PRS5 silencing (➀, ➁, and ➂). The phosphorylation of AKT and C-Fos was detected by Western-blot assay. As shown in **Figure 4D**, RANKL induction significantly promoted the phosphorylation of the key protein in PI3K/ATK and MAPK pathways AKT and C-Fos (➁ vs. ➀, ➄ vs. ➃, *P* < 0.01); the M54 treatment ameliorated the effects of RANKL induction (➂ vs. ➁, ➄ vs. ➅, *P* < 0.01); the RPS5 silencing blocked the effects of M54 (➅ vs. ➂, *P* < 0.01); the blockage of RPS5 silencing on M54’s effect was partially (➅ vs. ➄ and ➂ vs. ➁, *P* < 0.01).

### RPS5 Silencing Partially Ameliorates the Effects of M54 on Osteoclastogenesis-Related Markers Expression

The effect of RPS5 to osteoclastogenesis-related markers expression was also investigated with Western-blot assay. Two series of experiments with RANKL induction and M54 (1 μM) treatment were conducted in both cells with RPS5 silencing (➃, ➄, and ➄) or without PRS5 silencing (➀, ➁, and ➂). As shown in **Figure 5**, RANKL induction significantly promoted the expression of Cathepsin K, CTR, MMP-9, NFATc1, and TRAP (➁ vs. ➀, *P* < 0.01); the M54 treatment ameliorated the effects of RANKL induction (➃ vs. ➁, *P* < 0.01); the RPS5 silencing blocked the effects of M54 (➄ vs. ➃, *P* < 0.01); the blockage of RPS5 silencing on M54’s effect was partially (➄ vs. ➃, *P* < 0.01).

**FIGURE 5:** RPS5 regulates expressions of osteoclastogenesis-related markers. Western blot and optical density analysis of expression of Cathepsin K, CTR, MMP-9, NFATc1, and TRAP with Beta actin as reference. ➀RAW264.7 cells; ➁RAW264.7 induced with M-CSF, RANKL and PBS; ➂RAW264.7 cells infected with Lv-shRNA-RPS5 and induced with M-CSF, RANKL and PBS; ➃RAW264.7 cells induced with M-CSF, RANKL and treated with 4 μM M54; ➄RAW264.7 cells infected with Lv-shRNA-RPS5, induced with M-CSF, RANKL and treated with 4 μM M54. The membranes were cut according to the molecular size of the target protein and reincubated with primary antibodies but using the same loading control (^∗∗^*P* < 0.01, ^∗^*P* < 0.05 vs. ➁).

### M54 Inhibits Ovariectomy-Induced Bone Loss *in Vivo*

The OVX mouse was used to explore whether M54 can prevents post-menopause bone loss. Histological analysis included H&E staining (**Figure 6A**) and TRAP staining (**Figure 6B**). OVX significantly (*P* < 0.01) promoted trabecular bone loss, and M54 treatment prevented the change (**Figure 6A**). Osteoclasts were increased in OVX group, and M54 treatment ameliorated the increase (**Figure 6B**). The results were confirmed by Micro-CT results, which includes the two-dimensional structure and three-dimensional structure and the BV/TV, BS/TV, Tb.N, and BMD parameters statistics (**Figures 6C,D**). Consistent with this, the serum levels of TRAcp5B, IL-6, and TNF-α induced by OVX were also reduced by M54 treatment (**Figure 6E**).

**FIGURE 6:** M54 prevents ovariectomy-induced bone loss *in vivo*. **(A)** Representative H&E staining of distal femoral sections and quantification of trabecular area from each group 6 week after the operation (×40). **(B)** Representative TRAP-stained histologic distal femur sections from sham, OVX and OVX + M54 group (×400). **(C)** Micro CT analysis of the distal femur from sham, OVX, and OVX + M54 group. **(D)** Calculations of bone value/total value (BV/TV), trabecular number (Tb.N), bone mineral density (BMD), and bone surface area/total value (BS/TV). **(E)** Serum TRAcp5B, TNF-α, and IL-6 were examined (^∗^*P* < 0.05, ^∗∗^*P* < 0.01, ^∗∗∗^*P* < 0.001).

## Discussion

In this study, we demonstrated that M54 effectively prevented RANKL induced osteoclastogenesis *in vitro* and ovariectomy-induced bone loss *in vivo*. By now, this is the first study to demonstrate the effects of M54 on bone metabolism. We found that M54 inhibited bone loss *in vivo* and decreased the serum level of TRAcp5B. Besides M54 inhibited multiple pathways downstream of RANKL, including NF-κB, MAPK, and AKT pathways. Silencing RPS5 could prevent the inhibiting effects of M54 on RANKL induced pathways. These results indicated that M54 may be combined with RPS5 to inhibit osteoclastogenesis (**Figure 7**). And the results of alizarin red staining showed that there was no significant difference on osteogenesis after M54 treatment (**Supplementary Figure S1**). These results indicated that the main mechanism of M54 to reduce ovariectomy induced bone loss is to inhibit RANKL-induced osteoclastogenesis.

**FIGURE 7:** A schematic diagram which describes the mechanism that M54 inhibits RANKL-induced osteoclastogenesis. RANKL-RANK signaling induces NFATc1 expression through NF-κB, MAPKs, and PI3K/AKT pathways. M54 acts on the RPS5 and blocks NF-κB, MAPKs, and PI3K/AKT pathways and, subsequently, suppresses NFATc1 expression.

Over-activation of osteoclastogenesis and excessive osteoclastic bone resorption result in pathologic bone loss in diseases, including PMOP, RA, periodontitis, lytic bone metastasis, and Paget disease (Wang et al., 2012; Warren et al., 2015; Liu Q. et al., 2016). The osteoclasts’ resorption of bone in pathologic conditions (Krzeszinski et al., 2014), and RANKL activating downstream pathways including NF-κB, AKT, and MAPK (Asagiri and Takayanagi, 2007; Tao et al., 2016) are critical for the development of PMOP. Thus, inhibition of osteoclastogenesis is possibly effective for osteoporosis treatment (Anastasilakis et al., 2015; Arun et al., 2016; Feng et al., 2016). At the same time, inflammation plays a central role in the osteoclasts differentiation (Kikuta and Ishii, 2013; Liu Q. et al., 2016; Jordan et al., 2017). In PMOP, with the loss of estrogen, a potent inflammation inhibitor, the pro-inflammatory cytokines (TNF-α and IL-6) were increased and contributed to osteoclastogenesis by activating RANKL induced pathways (Lacativa and de Farias, 2010; Huang et al., 2016). And we observed that the serum level of IL-6 and TNF-α were increased in ovariectomized mice. These results indicated that inflammation contributed to osteoclastogenesis and bone resorption (Silverman et al., 2011; Vassalle and Mazzone, 2016). Thus, inhibiting osteoclastogenesis through anti-inflammation was a possible way to treat the PMOP.

Traditional Chinese medicine provided abundant resources for anti-osteoporosis drugs selection (Feng et al., 2017; Mei et al., 2017). In previous study, matrine, extracted from the sophora genus plants, was demonstrated to have a variety of pharmacological effects (Liu J. et al., 2016; Zhu et al., 2016). In our previous study, matrine derivative (M19) protected liver fibrosis by targeted to RPS5 in hepatic stellate cells (HSCs) and RPS5 overexpression in HSCs resulted in activation of AKT pathway (Xu et al., 2014). In this study, we synthesized the M54 based on the M19. M54 showed better anti-inflammatory activity and less cytotoxicity than M19. The MTT analysis showed that at the 100 μM concentration, the cytotoxic effect of M19 was 70% and M54 was 53% (**Supplementary Figure S2**). *In vitro* studies, the osteoclastogenesis experiment showed that at the 4 μM concentration of M19 and M54, the inhibiting osteoclastogenesis effect of M54 was more significant than M19 (**Supplementary Figure S3**). *In vivo* studies, the maximum tolerance dose of M54 for mice in this study was 250 mg/Kg and the value of M19 was 200 mg/Kg. In animal experiments, the levels of TNF-α and IL-6 of mice treated with M54 were significantly lower than those treated with M19. For further research, we performed experiment *in vitro* to investigate the effects of M54 on osteoclastogenesis and osteoclast function and investigated the signaling mechanisms in that process.

This study also showed that M54 inhibited OVX-induced bone loss by H&E staining of the distal femur and Micro-CT. And M54 inhibited osteoclastogenesis around the trabecular bone observed by TRAP staining. At the same time, bone resorption experiments *in vitro* also showed that M54 also inhibited the osteoclasts function. To clarify the mechanism of M54 effects on osteoclastogenesis, we performed the pre-experiment and selected the 1, 2, and 4 μM M54 for *in vitro* studies. M-CSF and RANKL induced the BMMCs and RAW264.7 cells to osteoclasts. M54 inhibited differentiation of pre-osteoclast into osteoclasts induced by RANKL, and it indicated that M54 blocked osteoclastogenesis. RANKL activated downstream pathways in the process of osteoclastogenesis including NF-κB, AKT, and MAPK pathways (Kaminski et al., 2015). As is well-known, RANKL binds to RANK and then activates the NF-κB pathway (Feng et al., 2014). For the AKT and MAPK pathways, the well-known activated protein kinases are AKT, ERK, JNK, and P38 (Guan et al., 2015; Asati et al., 2016; Tao et al., 2016). In our study, M54 inhibited expression of the key factors including AKT (PI3K/AKT pathway), P65, IκB (NF-κB pathway), ERK, JNK, P38 (MAPK pathway). Besides, the expression of NFATc1 was also inhibited.

Based on previous reports, the TRAP, Cathepsin K, TRAF6, CTR, and MMP9 were selected as osteoclastogenesis-related markers in this study (Kamiya et al., 1998; Li et al., 2011; Wu et al., 2012). And we clarified that M54 also inhibited the expression of MMP-9, TRAP, C-Src, and Cathepsin K.

According to our former study (Xu et al., 2014), another kind of matrine derivative (M19) could bind and stabilize RPS5, subsequently protected liver fibrosis in HSCs. And it was demonstrated that the mechanism of RPS5’s effects was to regulate Akt pathway (Xu et al., 2014). In this study, M54 exhibited more affinity to RPS5 and less cytotoxicity than M19. And in the present experiment, it was proved that M19 had the inhibitive effect on osteoclastogenesis. Thus, we hypothesized that RPS5 was related to M54’s effects on osteoclastogenesis, and we hypothesized that the mechanism was that M54 treatment stabilized RPS5. After induction, the RPS5 level was decreased possibly through ubiquitination, the mechanism of M54’s effect on RPS5 was to bind to and stabilize RPS5, thus M54 treatment could keep the RPS5 level and the relate signal transduction after induction.

The subsequent experiments showed that RPS5 level was significantly decreased during osteoclastogenesis, and was partially restored by M54 treatment. RPS5 silencing drastically compromised the inhibitory effects of M54 on osteoclastogenesis. And the expression of osteoclastogenesis-related markers was elevated by RPS5 silencing. The above results indicated the important role of RPS5 in osteoclastogenesis. The signaling mechanism was also explored. Besides the proved Akt pathway, the MAPK, and NF-κB pathways were also observed to be up-regulated by RPS5 silencing. At the same time, M54 treatment partially inhibited the activation of these pathways. The present experiment for the first time revealed the new function of RPS5 on osteoclastogenesis, and the mechanism was related to Akt, MAPK, and NF-κB pathways.

Although there have been increasing evidences proving the extraribosomal functions of RPS5 (Joseph et al., 2014; Bhat et al., 2015), however the mechanism has not been explained yet. It was demonstrated that Akt pathway could be regulated by RPS5, however, the exact role of RPS5 of the multiple cell signaling pathways, such as NF-κB, MAPK pathways has not been investigated before. For the first time, our study demonstrated that the expression of RPS5 significantly affected osteoclastogenesis, which indicated that RPS5 was promisingly the candidate target for primary osteoporosis treatment. Besides the major role which RPS5 played on Akt pathways, we also for the first time observed the regulation effect of RPS5 on NF-κB, MAPK pathways. According to the above results, we could confirm the important role of RPS5 in intracellular cell signaling transduction. However, the exact mechanism of RPS5 affecting the signaling pathways remains to be clarified in the future research.

There are still two limitations in our study. Firstly, in this study we confirmed the role of RPS5 in the process of osteoclastogenesis and the development of PMOP. However, the exact RPS5 related mechanisms in osteoporosis still need to be researched. Secondly, although we confirmed that the Chinese herb derivative M54 had significant effect to prevent the development of PMOP. However, there’s still a long way for us to take M54 into clinical use. Future clinical trials of M54 need to be conducted.

This study uncovered the key role of RPS5 in the development of osteoporosis. M54 was successfully synthesized and proved targeted to RPS5, exhibiting significant inhibitory effects on osteoclastogenesis by suppressing RANKL induced NF-κB, PI3K/AKT, and MAPK pathways activation and the expression of NFATc1 *in vitro*. And *in vivo* studies indicated that M54 could prevent ovariectomy-induced osteoporosis. In conclusion, RPS5 plays a key role in osteoclastogenesis and is a promising pharmaceutical target for PMOP.

## Author Contributions

CX, ZXin, and SJ designed this study; ZXin, CJ, and ZZ finished the animal studies and BMMCs isolation; WW, QL, ZXia, CL, and PP performed Western blotting; HH, ZQ, and LC synthesized M54.

## Conflict of Interest Statement

The authors declare that the research was conducted in the absence of any commercial or financial relationships that could be construed as a potential conflict of interest. The reviewer AR and the handling Editor declared their shared affiliation.

## Supplementary Material

FIGURE S1 M54 can not inhibits osteogenesis *in vitro*.

FIGURE S2 M54 showed less cytotoxicity than M19.

FIGURE S3 The inhibiting osteoclastogenesis effect of M54 was more significant than M19.
